# Adaptive double threshold energy detection based on Markov model for cognitive radio

**DOI:** 10.1371/journal.pone.0177625

**Published:** 2017-05-16

**Authors:** Yulei Liu, Jun Liang, Nan Xiao, Xiaogang Yuan, Zhenhao Zhang, Meng Hu, Yulong Hu

**Affiliations:** 1 Institute of Information and Navigation, Air Force Engineering University, Xi’an, Shanxi, China; 2 PLA stationed in Reserve Training Office of Lanzhou University, Lanzhou Jiaotong University, Lanzhou, Gansu, China; Universidad de Salamanca, SPAIN

## Abstract

The rapid development in the area of cognitive radio technology leads the society to higher standards of spectrum sensing performance, particularly in low signal-to-noise ratio (SNR) environment. This article proposes an adaptive double-threshold energy sensing method based on Markov model (ADEMM). When using the double-threshold energy sensing method, the modified Markov model that accounts for the time varying characteristic of the channel occupancy was presented to resolve the ‘confused’ channel state. Furthermore, in order to overcome the effect of noise uncertainty, the findings of this article introduce an adaptive double-threshold spectrum sensing method that adjusts its thresholds according to the achievable maximal detection probability. Numerical simulations show that the proposed ADEMM achieves better detection performance than the conventional double-threshold energy sensing schemes, especially in very low SNR region.

## Introduction

Recent decades witnessed a dramatic increase in the number of wireless communication users. Available spectrum resources are lacking without efficient management. According to Federal Communications Commission’s (FCC) recent study report [1], the assigned spectrum is not being fully utilized at a specific time and at particular geographic location resulting in a lot of underutilized spectrum resources. Cognitive radio (CR) is a key enabling technology which effectively provides the capability to used underutilized part of the spectrum and serves it as a remedy for plausible spectrum shortage problem. In the CR-based system, the secondary user (SU) exploits the spectrum opportunity, which is defined as the frequency channel that is temporarily not used by the primary users (PUs) [2]. CR which includes spectrum sensing, spectrum accessing, power control and intelligent management is widely used in a new generation of wireless communication system [3]. Therefore, as a key technique in the CR system, spectrum sensing recently gained much attention in the researching area and its development played and will continue to have a significant role in promoting CR realization.

Several techniques advocated for spectrum sensing, which includes energy sensing, coherent sensing, cyclostationarity-based sensing, autocorrelation sensing, radio identification, and some other methods (multi-taper estimation, wavelet transforms, Hough transform, and time-frequency analysis) [4–6]. Among aforementioned spectrum sensing techniques, energy sensing became the most commonly-used method since it is simple and it does not require prior knowledge of the PUs’ signals, which results in simple implement. However, traditional energy sensing method does not make a good performance under low SNR. Different from the conventional energy detection using single threshold, some works started to take double thresholds judgment into consideration recently [7–11]. In Ref [7], a new cooperative spectrum sensing scheme based on two-stage detectors was proposed, which chose single threshold during the first stage and double-threshold in the second stage. Another two-step spectrum sensing scheme to improve detection performance was put forward in Ref [8], which consists of two sensing methods, respectively, double-threshold energy sensing in the first step and cyclostationarity-based sensing in the second step. However, it is computationally complex and requires longer sensing time. In Ref [9], a double-threshold method is applied to perform spectrum sensing, while the local energy detection results are divided into a hard decision and soft decision. Since the final decision is made by the fusion center, this collaborative method is difficult to implement. In Ref [10], the author maximizes the throughput of a cooperative CR network by optimizing the parameter *k* in a *k*-out-of-*n* fusion rule, while sensing thresholds were kept constant during that period. In Ref [11], the spectrum sensing process is divided into several stages. When the energy value falls between two thresholds, which are varied based on the number of samples, the CR will move to the next stage to collect more samples until the decision can be made. However, sometimes in order to reach a conclusion, the stages would be repeated again and again. As a result, the timeliness of the sensing will be accordingly decreased.

However, to the best of our knowledge, all the above mentioned sensing schemes have successfully avoided the problem of calculating the double-threshold. Although some of them introduced noise uncertainty to calculate the double-threshold, the noise uncertainty is still unknown in the real environment. Secondly, a majority of the double-threshold energy sensing methods have been used in the cooperative environment or with the other sensing schemes, which will increase the computational complexity and sensing time. On the other hand, there is no further description about the performance of sensing time which has a significant impact over spectrum sensing.

This paper introduces an adaptive double—threshold energy sensing algorithm for CR. In the proposed approach, the energy sensing algorithm adapts its double-threshold based on the optimal function within the constraint condition. In addition, we also set up a novel spectrum occupancy model based on a two Markov chain. If the received signal energy is greater than the upper bound threshold, the channel will be declared to be occupied; if the decision metric is below the lower bound threshold, the channel will be declared to be empty and available for SU; if the collected energy value falls between the two thresholds, the channel state will be judged by the statistic previous channel states. In addition, mathematical expressions for the probability of detection and the probability of false alarm are also derived.

In Section II, an introduction to the algorithm of double-threshold energy sensing is provided. Section III presents details on the Markov model of spectrum occupancy. Section IV describes the adaptive double-threshold processing. The proposed scheduling algorithm is discussed in Section VI followed by numerical simulation results. Section VII concludes the manuscript.

## Energy sensing

It is assumed that the wideband frequency range is divided into *K* sub-channels each with the same bandwidth, where a sub-channel is in a portion of spectrum is defined at a certain frequency *f*_*i*_. We consider the problem of detecting the presence of one PU at a given sub-channel based on the signal observed by the SU. Therefore, this is a binary hypothesis problem. In the *i*-th sub-channel *f*_*i*_, we can use the following hypothesis for the received signal *r*_*i*_(*m*) of the *m*-th sampling results [12, 13]:

$$r_{i}(m)=\{\begin{array}{c} w_{i}(m),\;H_{0}\\ s_{i}(m)h_{i}(m)+w_{i}(m),\;H_{1} \end{array}$$ (1)

where *s*_*i*_(*m*) is the PU licensed signal in the *i*-th sub-channel *f*_*i*_ (*i* = 1, 2,…, *K*; *m* = 1, 2,…, *M*), $w_{i}(m)∼N(0,\sigma_{w}^{2})$ is additive white Gaussian noise with zero mean and variance $\sigma_{w}^{2}$, and *h*_*i*_(*m*) denotes the Rayleigh fading channel gain of the sensing channel between the PU and the SU. *H*_0_ is a null hypothesis, which indicates the absence of PU(band free), and *H*_1_ is the alternative hypothesis, which implies that PU is present(band occupied).

### Conventional energy sensing

In the conventional energy sensing, the SU makes its local decisions by comparing its observation with a pre-fixed threshold.

A sub-channel is either free (*H*_0_) or occupied by a PU (*H*_1_). Decision *H*_0_ or *H*_1_ will be made when the energy of the PU signal in this sub-channel is less or greater than the threshold value *V*_*th*_, respectively. The test statistic is given by [14]

$$R=\frac{1}{N}\sum_{n=1}^{N}{\left|r_{i}(m)\right|}^{2}$$ (2)

where *r*_*i*_(*m*) is the received input signal, *N* is the number of samples, and *R* denotes the energy of the received input signal.

When *N* of energy sensing is very large and the received signal *r*_*i*_(*m*) are independent, the test statistic *R* in a sub-channel can be approximated as a normal variable. As a result, *R* follows a normal distribution under *H*_0_ and *H*_1_:

$$R∼\{\begin{array}{ll} N(\sigma_{w}^{2},\frac{2\sigma_{w}^{4}}{N}) & H_{0}\\ N(\sigma_{w}^{2}+\sigma_{s}^{2},\frac{2{\left(\sigma_{w}^{2}+\sigma_{s}^{2}\right)}^{2}}{N}) & H_{\text{1}} \end{array}$$ (3)

where $\sigma_{w}^{2}$ and $\sigma_{s}^{2}$ are the noise variance and signal variance, respectively.

Threshold value is set to meet the target probability of false alarm *P*_*f*_ according to the noise power. The probability of detection *P*_*d*_ and the probability of missing *P*_*m*_ can also be identified. The expression for *P*_*f*_, *P*_*d*_ and *P*_*m*_ can be formulated as [15]

$$\begin{array}{ll} P_{f}=P\left\{R>V_{th}|H_{0}\right\} & =Q\left(\frac{V_{th}-N\sigma_{w}^{2}}{\sqrt{2N\sigma_{w}^{4}}}\right)\\ & =Q\left(\sqrt{\frac{N}{2}}(\frac{V_{th}}{N\sigma_{w}^{2}}-1)\right)\\ & =Q\left(\sqrt{\frac{N}{2}}({\tilde{V}}_{th}-1)\right) \end{array}$$ (4)

$$\begin{array}{ll} P_{d}=P\left\{R>V_{th}|H_{1}\right\} & =Q\left(\frac{V_{th}-N(\sigma_{w}^{2}+\sigma_{s}^{2})}{\sqrt{2N{\left(\sigma_{w}^{2}+\sigma_{s}^{2}\right)}^{2}}}\right)\\ & =Q\left(\sqrt{\frac{N}{2}}\frac{V_{th}/(N\sigma_{w}^{2})-(1+\gamma )}{1+\gamma }\right)\\ & =Q\left(\sqrt{\frac{N}{2}}\frac{{\tilde{V}}_{th}-(1+\gamma )}{1+\gamma }\right) \end{array}$$ (5)

$$P_{m}=P\left\{R<V_{th}|H_{1}\right\}=1-P_{d}$$ (6)

where *Q*(·) denotes Gaussian tail probability *Q*-function, $\gamma =\sigma_{s}^{2}/\sigma_{w}^{2}$ represents the SNR of each sub-channel. Let ${\tilde{V}}_{th}=V_{th}/(N\sigma_{w}^{2})$, then, from Eqs (4) and (5), it is observed that *P*_*f*_ is independent of ${\tilde{V}}_{th}$, and *P*_*d*_ is a function of ${\tilde{V}}_{th}$ for given *γ* and *N*.

### Double-threshold energy sensing

Generally it is assumed that noise power in the receiver attains a certain level. Practically, noise is not only limited to Gaussian White Noise, in fact, it is a sum of various other factors as well. Thus, noise power changes within limits with passage of time and relative location, this phenomenon is referred to as ‘noise uncertainty’. It is often the case that the received signal cannot be distinguished due to dynamically changing noise power. As a result, detection performance degrades i.e., the probability of detection decreases and probability of false alarm increases, particularly when the range of noise uncertainty increases. Thus, double-threshold energy sensing method is being proposed which makes the detection result more reliable and minimizes the influence of so called noise uncertainty.

Noise uncertainty as discussed in [16]:

$$\rho =\frac{{\hat{\sigma }}_{w}^{2}}{\sigma_{w}^{2}}\in \left[10^{-A/10},10^{A/10}\right],A\geq 0$$ (7)

where ${\hat{\sigma }}_{w}^{2}$ is a real noise variance, *A* is the maximum noise uncertainty and upper bounded by 10lg *ρ*, and size of 10lg *ρ* is uniformly distributed over the interval [−*A*, *A*].

Therefore, noise uncertainty defines the lower threshold *V*_*th*1_ and the upper threshold *V*_*th*2_:

$$V_{th1}=\left(\sqrt{\frac{2}{N}}Q_{}^{-1}\left(P_{f}\right)+1\right)\frac{1}{\rho }\sigma_{w}^{2}$$ (8)

$$V_{th2}=\left(\sqrt{\frac{2}{N}}Q_{}^{-1}\left(P_{f}\right)+1\right)\rho \sigma_{w}^{2}$$ (9)

Conventionally, the state of a specific sub-channel is classified by two random variables (RVs), i.e., ‘band occupied’ (signal present) and ‘band free’ (signal absent) [7]. However, sometimes the sub-channel state can be referred to as ‘confused’. The two thresholds *V*_*th*1_ and *V*_*th*2_ classify the test statistic *R* in a sub-channel into primary signal (represented as ‘1’), noise (represented as ‘0’), or confused (represented as ‘*x*’) state:

$$R_{c}=\{\begin{array}{lll} 1 & R>V_{th2} & H_{1}\\ x & V_{th1}\leq R\leq V_{th2} & H_{}\\ 0 & R<V_{th1} & H_{0} \end{array}$$ (10)

where *R*_*c*_ is a occupancy state of a sub-channel. Fig 1 illustrates the three states of a sub-channel, where confused region is bounded by the area between *V*_*th*2_ and *V*_*th*1_. In this region, the detection between the noise and PU signal cannot be optimally obtained using single threshold.

**Fig 1:** Illustration of energy distribution of PU and noise signals.

To rectify the problem of ‘confused’ state, some scholars use other detection methods, such as the cyclostationarity of PUs’ signal is exploited in [8], the additional information or collaboration of a receiver with other radios in the network is employed in [17], covariance detection is utilized in [18]. Here, based on the advantages of listen-before-talk, we set up a Markov Model based on time-varying parameters for spectrum occupation to resolve this is called confused state.

## Markov model based on time-varying parameters for spectrum occupancies

This section we present a statistical approach to efficiently develop Markov models which could be employed to model both stationary as well as non-stationary spectrum occupancies.

### Markov model

The primary channel is assumed as a time division multiple address (TDMA) operating manner. The activity of the PU is assumed to be characterized by a two-state Markov channel with transition probabilities *P*_10_, from free to occupied, and *P*_01_, from occupied to free. At the beginning of each slot, SU senses the channel to acquire the opportunity for accessing.

As shown in Fig 2, the two state Markov chain model is enough to classify the occupancy state of a sub-channel. The parameters of Markov model are the state probabilities denoted as *P*_0_ and *P*_1_ corresponding to the states 0 and 1, respectively, and the state transition probabilities are represented as *P*_00_, *P*_01_, *P*_10_, *P*_11_. In previous works [19–21], it was assumed that when building a Markov model for the channel occupancy, the channel occupancy is stationary or divided into several stages, whereas, in practice, the model parameters may vary with time. For instance, the utilization of a cellular mobile channel varies drastically in different instances of the day with peak usage during business hours. Therefore, to compute the model parameters, a weighted approach is employed, where the current and most recent instantaneous channel state is heavily weighted.

**Fig 2:** Channel state’s Markov model.

### Time-varying parameters estimation

To keep a track of dynamically changing time varying channel occupancy, we present a weighted scheme, where higher weight is assigned to the current and most recent instantaneous channel state.

At a particular time instant *t*_*k*_ and for the *i*-th sub-channel the weight count of past occurrences of state 1 is determined by *R*_*c*_, denoted as $N_{c}(R_{c,t_{j}}=1)$, and the corresponding weighted state probability is defined as,

$$P_{1}^{i}(t_{k})=\frac{N_{c}(R_{c,t_{j}}=1)}{N_{t_{k}}}\;j=1,2,\ldots ,k$$ (11)

The assigned weights depend on the occurrence time of the channel state relative to *t*_*k*_, where *t*_*k*_ is a discrete time variable, and the total number of measurement samples collected from time *j* = 1 to *k* is denoted as $N_{t_{k}}$. The estimate of the true probability $P_{1}^{i}(t_{k})$ is obtained from the finite set of spectrum measurement samples using

$${\bar{P}}_{1}^{i}(t_{k})=\frac{\sum_{j=1}^{k}R_{c,t_{j}}\cdot \text{exp}\left(\eta (t_{k}-t_{j})\right)}{N_{t_{k}}}$$ (12)

where *η* is the forgetting factor for 0 ≤ *η* ≤ 1 and is employed to give more weight to the most recent samples and less weight to previous samples. Similarly, the *i*-th sub-channel state transition probability $P_{01}^{i}$ is determined as,

$${\bar{P}}_{01}^{i}(t_{k})=\frac{N_{c}(R_{c,t_{j+1}}=1,R_{c,t_{j}}=0)}{N_{t_{k}}-1}\;j=1,2,\ldots ,k-1$$ (13)

The remaining model parameters can be determined in a similar way.

To derive the sampling distribution for the model parameters it is assumed that the channel occupancy is piecewise stationary. For instance, during the non-peak hours on a normal weekday, the channel occupancy in a cellular mobile band is less and remains approximately stationary. In our discussion, we assume that the channel occupancy is stationary over a particular period of time.

In order to estimate the parameters of the channel state, it is assumed that *R*_*c*_ is ergodic and the samples are independent. Moreover, since the state occupancy is assumed to be piecewise stationary, we determine the parameters of the state over a segment of time. Then the $N_{t_{k}}$ constitutes the sample space of *R*_*c*_. If *T* is the total time duration and Δ*t* is the time spacing, then $T=N_{t_{k}}\cdot \Delta t$.

The true probability $P_{1}^{i}$ of the state occupancy, which is also a mean occupancy in the *i*-th sub-channel is estimated as,

$${\bar{P}}_{1}^{i}=\frac{\sum_{j=1}^{t_{k}}R_{c,t_{j}}}{N_{t_{k}}}$$ (14)

$${\bar{\sigma }}_{s}^{2}=\frac{\sum_{j=1}^{N_{t_{k}}-1}{\left(R_{c,t_{j}}-{\bar{P}}_{1}^{i}(t_{k})\right)}^{2}}{N_{t_{k}}-1}$$ (15)

In Eq (14), $R_{c,t_{j}}$ represents samples of the two state RVs and summation of the samples, which is the number of instances when the channel is occupied, followed by a binomial distribution $B(N_{t_{k}},P_{1}^{i})$. ${\bar{P}}_{1}^{i}$ is a consistent estimator of $P_{1}^{i}$ which can be treated as a RV with a certain sampling distribution. For large $N_{t_{k}}^{}$($N_{t_{k}}^{}>100$), the binomial distribution can be approximated with a normal distribution. Thus ${\bar{P}}_{1}^{i}$ can be considered as a Gaussian RV with normalized form denoted as z ~ N(0, 1). If *α* is the confidence coefficient, we can denote the 100*α* percentage point by *z*_*α*_ [22]. Let *t*_*n*_ be the corresponding RV with a student *t* distribution of *n* (*n* = *N* − 1) degrees of freedom and is 100*α* percentage point is denoted as *t*_*n*, *α*_. From the sampling distribution of ${\bar{P}}_{1}^{i}$, the confidence interval for $P_{1}^{i}$ can be defined as [23]

$$\text{Prob }\left[{\bar{P}}_{1}^{i}-d\leq P_{1}^{i}\leq {\bar{P}}_{1}^{i}+d\right]=1-\alpha ,\;d=\frac{{\bar{\sigma }}_{s}t_{n,\alpha }}{\sqrt{N_{t_{k}}}}$$ (16)

From Eq (16) it is observed that for a given confidence interval, the estimated accuracy increases with a proportional increase in the number of samples $N_{t_{k}}$.

### Listen-before-talk scheme

In conventional ED-based spectrum sensing, noise uncertainty increases the difficulty in setting the optimal threshold for a CR and thus degrades its sensing reliability. In addition, this may not be optimum in low-SNR conditions where the performance of fixed single threshold (*γ*)-based detector can vary from the targeted performance metrics substantially. In order to overcome the defects of fixed single threshold-based detector, the double threshold-based detector emerges as the times require.

In Fig 1, the area comes under lower bound (*λ*_1_) and upper bound (*λ*_2_) is known as confused region. In this region, the detection between noise and PU signal is difficult using single threshold. In the proposed ADEMM scheme, the lower bound threshold (*λ*_1_) and the upper bound threshold (*λ*_2_) are selected according to the maximum probability detection. And both of the thresholds are given the analytical solution in section IV. Furthermore, the confused region is resolved by the Markov Model based on time-varying parameters. If the detected energy values (*R*) fall in the confused region, it will adopts the listen-before-talk mechanism, and are compared with transmission probability to make a final decision at a fixed probability of false alarm. If the values lie outside the confused region, it will generate 0 or 1 depending upon signal existence. Thus, the numerical results show that the proposed scheme enhances the detection performance.

The listen-before-talk scheme employs the knowledge of previously observed channel state and thus, resolves the ‘confused’ channel state. Fig 3 shows the process of resolving the confused state in the channel state. Furthermore, the decision over a threshold may also be based on the observation of the channel state over a specified period of time rather than only relying over a previous channel state.

**Fig 3:** Analysis of the channel state.

As in the case, if current channel state is observed to be ‘confused’, the current state is chosen based over the characteristic of the period channel state. When the previous channel state was ‘band occupied’, if $P_{11}^{i}(t_{k-1})>P_{10}^{i}(t_{k-1})$, then the current state is also declared to be ‘occupied’, otherwise it is declared to be ‘free’. When the previous channel state was ‘band free’, if $P_{01}^{i}(t_{k-1})>P_{00}^{i}(t_{k-1})$, then the current state is also declared to be ‘occupied’, otherwise it is declared to be ‘free’.

For false alarm probability *P*_*f*_ = 0.1, the confidence level is 95%. SNR range varies from -30 to 0dB and QPSK modulation is considered in AWGN channel. Fig 4 presents the performance comparison of the double threshold energy sensing based on Markov model (DEMM) under different noise uncertainty levels. It is observed that the noise uncertainty has a significant impact over the probability of detection. DEMM algorithm is less influenced by noise uncertainty in the -8dB which can be neglected. However, as SNR drops and noise uncertainty increases, the performance of DEMM rapidly drops. For example, when the noise uncertainty increases by 8.91% at -10dB, the performance of DEMM will be reduced by 67.1%. Especially, when the SNR approaches -12dB, with the increase of noise certainty, the performance of DEMM could not meet the requirement of detection. From Eqs (8) and (9), it can be seen that when *ρ* = +∞, *V*_*th*1_ = 0 and *V*_*th*2_ = +∞, which suggests that most of the test statistic *R* will be in the confused region. As a result, all of the judgment results depend on the previously observed channel states, that is to say, the current channel information cannot make a contribution to the judgment since the double threshold adjustment is not reasonable. Therefore, an adaptive double-threshold is proposed in order to rectify this artifact.

**Fig 4:** Performance comparison with different noise uncertainty levels.

## Adaptive double-threshold energy sensing

Based on the double-threshold sensing and Markov model of spectrum occupancy, we propose an adaptive double-threshold energy sensing method.

Let *P*_*f*_ denotes the probability of false alarm and *P*_*d*_ denotes the probability of detection. Then,

$$P_{f}=P\left\{R>V_{th2}|H_{0}\right\}+P\left\{V_{th1}\leq R\leq V_{th2}|H_{0}\right\}\cdot \left(P_{0}P_{01}+P_{1}P_{11}\right)$$ (17)

$$P_{d}=P\left\{R>V_{th2}|H_{1}\right\}+P\left\{V_{th1}\leq R\leq V_{th2}|H_{1}\right\}\cdot \left(P_{0}P_{01}+P_{1}P_{11}\right)$$ (18)

Since *R* follows a normal distribution under *H*_0_ and *H*_1_:

$$P\left\{R>V_{th2}|H_{0}\right\}=P_{f|V_{th}=V_{th2}},P\left\{R>V_{th1}|H_{0}\right\}=P_{f|V_{th}=V_{th1}}$$ (19)

$$P\left\{R>V_{th2}|H_{1}\right\}=P_{d|V_{th}=V_{th2}},\;P\left\{R>V_{th1}|H_{1}\right\}=P_{d|V_{th}=V_{th1}}$$ (20)

Then

$$P_{f}=P_{f|V_{th}=V_{th2}}+(P_{f|V_{th}=V_{th1}}-P_{f|V_{th}=V_{th2}})\cdot (P_{0}P_{01}+P_{1}P_{11})$$ (21)

$$P_{d}=P_{d|V_{th}=V_{th2}}+(P_{d|V_{th}=V_{th1}}-P_{d|V_{th}=V_{th2}})\cdot (P_{0}P_{01}+P_{1}P_{11})$$ (22)

According to the Neyman-Pearson criterion [17], the aim of a given probability of false alarm *β* is to get the optimal double-threshold, *V*_*th*1_ and *V*_*th*2_, such that the double-threshold jointly maximizes the probability of detection *P*_*d*_. The corresponding problems can be described as

$$\begin{array}{l} \underset{V_{th1},V_{th2}}{\text{max}}\;P_{d}(V_{th1},V_{th2})\\ \text{ s}.\text{t}.\;P_{f}=\beta \end{array}$$ (23)

From Eqs (17) to (20), the relationship between the thresholds, *V*_*th*1_ and *V*_*th*2_, can be described as

$$V_{th1}=f(V_{th2})$$ (24)

Furthermore, the problem in Eq (23) can be rewritten as

$$\underset{V_{th2}}{\text{max}}\;P_{d}(f(V_{th2}),V_{th2})$$ (25)

The optimal *V*_*th*2_ can be obtained from Eq (25). Then, the optimal *V*_*th*1_ can be obtained by substituting the optimal *V*_*th*2_ in Eq (24).

The detailed expressions for *P*_*d*_ and *P*_*f*_ can be obtained by substituting Eqs (4), (5) and (24) into Eq (22).

$$\begin{array}{l} P_{d}=Q\left(\sqrt{\frac{N}{2}}\frac{V_{th2}/(N\sigma_{w}^{2})-(1+\gamma )}{1+\gamma }\right)+(P_{0}P_{01}+P_{1}P_{11})\cdot \\ \;\left[Q\left(\sqrt{\frac{N}{2}}\frac{V_{th1}/(N\sigma_{w}^{2})-(1+\gamma )}{1+\gamma }\right)-Q\left(\sqrt{\frac{N}{2}}\frac{V_{th2}/(N\sigma_{w}^{2})-(1+\gamma )}{1+\gamma }\right)\right]\\ =Q\left(\sqrt{\frac{N}{2}}\frac{{\tilde{V}}_{th2}-(1+\gamma )}{1+\gamma }\right)+\mu \cdot \left[Q\left(\sqrt{\frac{N}{2}}\frac{{\tilde{V}}_{th1}-(1+\gamma )}{1+\gamma }\right)-Q\left(\sqrt{\frac{N}{2}}\frac{{\tilde{V}}_{th2}-(1+\gamma )}{1+\gamma }\right)\right]\\ =Q\left(\sqrt{\frac{N}{2}}\frac{{\tilde{V}}_{th2}-(1+\gamma )}{1+\gamma }\right)+\mu \cdot \left[Q\left(\sqrt{\frac{N}{2}}\frac{f({\tilde{V}}_{th2})-(1+\gamma )}{1+\gamma }\right)-Q\left(\sqrt{\frac{N}{2}}\frac{{\tilde{V}}_{th2}-(1+\gamma )}{1+\gamma }\right)\right] \end{array}$$ (26)

where ${\tilde{V}}_{th1}=V_{th1}/(N\sigma_{w}^{2}),\;{\tilde{V}}_{th2}=V_{th2}/(N\sigma_{w}^{2}),\;\mu =P_{0}P_{01}+P_{1}P_{11}$. In order to find the optimal ${\tilde{V}}_{th2}$ to maximize the probability of detection, the derivative of *P*_*d*_ is determined as

$$\begin{array}{ll} \frac{\partial P_{d}}{\partial {\tilde{V}}_{th2}} & =\sqrt{\frac{N}{\pi }}\cdot \frac{\mu -1}{2(1+\gamma )}\cdot \text{exp}\left(-\frac{N{\left({\tilde{V}}_{th2}-1-\gamma \right)}^{2}}{4{\left(1+\gamma \right)}^{2}}\right)-\sqrt{\frac{N}{\pi }}\cdot \frac{\mu }{2(1+\gamma )}\cdot \frac{\partial f({\tilde{V}}_{th2})}{\partial {\tilde{V}}_{th2}}\cdot \text{exp}\left(-\frac{N{\left(f({\tilde{V}}_{th2})-1-\gamma \right)}^{2}}{4{\left(1+\gamma \right)}^{2}}\right)\\ & =\sqrt{\frac{N}{\pi }}\cdot \frac{1}{2(1+\gamma )}\cdot \left[(\mu -1)\cdot \text{exp}\left(-\frac{N{\left({\tilde{V}}_{th2}-1-\gamma \right)}^{2}}{4{\left(1+\gamma \right)}^{2}}\right)-\mu \frac{\partial f({\tilde{V}}_{th2})}{\partial {\tilde{V}}_{th2}}\cdot \text{exp}\left(-\frac{N{\left(f({\tilde{V}}_{th2})-1-\gamma \right)}^{2}}{4{\left(1+\gamma \right)}^{2}}\right)\right] \end{array}$$ (27)

Since *P*_*f*_ = *β*, then calculating the derivative at both sides,

$$\begin{array}{ll} \frac{\partial P_{f}}{\partial {\tilde{V}}_{th2}} & =\sqrt{\frac{N}{\pi }}\cdot \frac{\mu -1}{2}\cdot \text{exp}\left(-\frac{N{\left({\tilde{V}}_{th2}-1\right)}^{2}}{4}\right)-\sqrt{\frac{N}{\pi }}\cdot \frac{\mu }{2}\cdot \frac{\partial f({\tilde{V}}_{th2})}{\partial {\tilde{V}}_{th2}}\cdot \text{exp}\left(-\frac{N{\left(f({\tilde{V}}_{th2})-1\right)}^{2}}{4}\right)\\ & =\frac{1}{2}\sqrt{\frac{N}{\pi }}\cdot \left[(\mu -1)\cdot \text{exp}\left(-\frac{N{\left({\tilde{V}}_{th2}-1\right)}^{2}}{4}\right)-\mu \cdot \frac{\partial f({\tilde{V}}_{th2})}{\partial {\tilde{V}}_{th2}}\cdot \text{exp}\left(-\frac{N{\left(f({\tilde{V}}_{th2})-1\right)}^{2}}{4}\right)\right]\\ & =0 \end{array}$$ (28)

From Eq (28), the $\frac{\partial f({\tilde{V}}_{th2})}{\partial {\tilde{V}}_{th2}}$ can be determined as,

$$\frac{\partial f({\tilde{V}}_{th2})}{\partial {\tilde{V}}_{th2}}=\frac{\mu -1}{\mu }\cdot \text{exp}\left(\frac{N(f({\tilde{V}}_{th2})+{\tilde{V}}_{th2}-2)\cdot (f({\tilde{V}}_{th2})-{\tilde{V}}_{th2})}{4}\right)$$ (29)

The derivative of *P*_*d*_ can be rewritten by substituting Eq (29) into Eq (27) as

$$\frac{\partial P_{d}}{\partial {\tilde{V}}_{th2}}=\sqrt{\frac{N}{\pi }}\cdot \frac{\mu -1}{2(1+\gamma )}\cdot \left[\text{exp}\left(-\frac{N{\left({\tilde{V}}_{th2}-1-\gamma \right)}^{2}}{4{\left(1+\gamma \right)}^{2}}\right)-\text{exp}\left(\frac{N(f({\tilde{V}}_{th2})+{\tilde{V}}_{th2}-2)\cdot (f({\tilde{V}}_{th2})-{\tilde{V}}_{th2})}{4}-\frac{N{\left(f({\tilde{V}}_{th2})-1-\gamma \right)}^{2}}{4{\left(1+\gamma \right)}^{2}}\right)\right]$$

Let $\frac{\partial P_{d}}{\partial {\tilde{V}}_{th2}}=0$, the only solution (assume ${\tilde{V}}_{th1}\neq {\tilde{V}}_{th2}$) of the equation can be computed as

$$f({\tilde{V}}_{th2})=\frac{2(\gamma +1)}{\gamma +2}-{\tilde{V}}_{th2}$$ (30)

Then ${\tilde{V}}_{th2}$ can be calculated by substituting Eq (29) into Eq (27) as

$${\tilde{V}}_{th2}=\frac{\gamma +1}{\gamma +2}+\frac{\gamma +2}{N}\text{ln}\frac{\mu }{1-\mu }$$ (31)

Then

$${\tilde{V}}_{th1}=f({\tilde{V}}_{th2})=\frac{2(\gamma +1)}{\gamma +2}-{\tilde{V}}_{th2}=\frac{\gamma +1}{\gamma +2}-\frac{\gamma +2}{N}\text{ln}\frac{\mu }{1-\mu }$$ (32)

**Algorithm 1**. Proposed adaptive double-threshold energy sensing algorithm.

For SUs

 Select the *i*-the sub channel of channel arranged in order of decreasing $P_{0}^{i}$

 Begin

 for *t*_*j*_ = 1,2,…,*T* do

  Perform local sensing and obtain $R_{t_{j}}$

  Set up the modified Markov model and calculate the parameters

  Set up objection function and obtain *V*_*th*1_, *V*_*th*2_

  if $0<R_{t_{j}}\leq V_{th1}$ then

   $R_{c,t_{j}}=0$

   Band available

  else if $V_{th2}\leq R_{t_{j}}$ then

   $R_{c,t_{j}}=1$

   Band occupied

  else employ the listen-before-talk approach

   if $R_{c,t_{j-1}}=1$ & $P_{11}^{i}(t_{j-1})>P_{10}^{i}(t_{j-1})$ then

    $R_{c,t_{j}}=1$

    Band occupied

   else if $R_{c,t_{j-1}}=0$ & $P_{01}^{i}(t_{j-1})>P_{00}^{i}(t_{j-1})$ then

    $R_{c,t_{j}}=1$

    Band occupied

   else

    $R_{c,t_{j}}=0$

    Band available

   End if

  End if

 End for

End

## Analysis of simulation experiment

In this section, we present numerical simulation results to verify the advantages of the proposed ADEMM spectrum sensing method.

In the following figures, we used the marker ‘DEMM’ to denote the DE-based on Markov model and “ADEMM” to denote the adaptive DE-based on Markov model. The cooperative spectrum sensing algorithm based on DE (CSBDE) is proposed by Ref [8] and the ‘Two-stage’ DE is suggested in Ref [7]. The two-step spectrum sensing scheme based on cyclostationarity (Cyclostationary-DE) is proposed by Ref [9] and the ‘VRODE’ is the method which is proposed in Ref [10]. The ‘ADE’ in Ref [11] is the adaptive double-threshold energy sensing algorithm. All the curves marked with ‘DE’ represent the double threshold energy sensing method. The ‘ME’ in Ref [21] is the single-threshold detector based on Markovian Estimation under the perfect knowledge performance bound.

The simulation setup is as follows: The PU signal is assumed to be a QPSK modulated signal *s*(*t*) = *A*_*m*_ cos(2*πf*_*i*_*t* + *ϕ*) = 0.3cos(2000*πt* + *ϕ*) after frequency mixing at the receiver in AWGN channel. The sampling frequency is *f*_*s*_ = 5MHz, and 1 − *α* = 0.95 with the confidence level being used to calculate the parameters of the Markov model for each decision making. Noise power estimation is conducted except for the cases where noise uncertainty is considered. The probability of false alarm is set to be *P*_*f*_ = 0.1.

Fig 5 shows the comparative performance of ADEMM under different noise uncertainty. It is seen that at SNR higher than -10dB, the performance of detection is hardly affected by noise uncertainty. When SNR is less than -10dB, the performance becomes poor with an increase in noise uncertainty. When SNR is -15dB, the detection performance decreases 2.73% with the noise uncertainty being increased to 8.91%. However, with the increase of noise uncertainty, especially when *ρ* > 1.1, the noise uncertainty results in a vital influence on the ADEMM algorithm. In contrast to Fig 4, it can be found that our proposed ADEMM spectrum sensing method is not sensitive to the common noise uncertainty. Thus, the proposed ADEMM is robust to noise uncertainty. The underlying reason lies in the fact that the double-threshold of ADEMM is calculated based on the maximal *P*_*d*_. Based on the above discussion, the optimal double-threshold can make most of statistics out the confused region under noise uncertainty.

**Fig 5:** Performance comparison with different noise uncertainty levels.

In Fig 6, the performance of the proposed scheme is compared with other existing schemes under the same noise uncertainty level *ρ* = 1.01. According to the simulation results, the proposed ADEMM is superior to other algorithms particularly when SNR is greater than -7dB. Although the performance of ADEMM, CSBDE, Cyclostationary-DE, “Two stage”-DE, VORDE, ADE and ME start to deteriorate at -15dB, -14dB, -11dB, -7dB, -12dB, -15dB and -9dB SNR, the ADEMM still improves detection performance and outperforms the CSBDE, Cyclostationary-DE, “Two stage”-DE, VORDE ADE and ME by 126%, 159%, 88%, 43%, 13% and 41% at SNR setting of as low as -20dB, respectively. It is further observed that the proposed spectrum sensing scheme achieves spectrum detection performance in the order of 0.9 for an SNR value of as low as -17dB. When the SNR falls between -7dB and -17dB, the detection performance of ADEMM and ADE is superior to the other algorithms since adaptive double-threshold improves the detection performance to a certain degree under low SNR. As the SNR continues to decrease, ADEMM proves better than the ADE which is due to the fact that the ‘listen before talk’ mechanism of ADEMM could further improve the detection performance of the confusion channel state. The performance of CSBDE(*N*_*r*_ = 2), Cyclostation-D VORDE(*N*_*r*_ = 2) and ME comes second. Although, the CSBDE(*N*_*r*_ = 2) collaborative detection algorithm can improve the detection performance to a certain extent, however, it cannot overcome the defects of double-threshold energy detection essentially. Cyclostation-DE algorithm solves the problem of confusion channel state by introducing the cycle stationary feature detection and thus the detection performance has made a certain improvement. VORDE(*N*_*r*_ = 2) maximizes the throughput of a cooperative CR network through optimizing the parameter *k* in a *k*-out-of-*n* fusion rule in order to improve the detection performance, However, since its sensing thresholds were kept constant, it could not make a good performance under low SNR circumstance. ME models correlation in PU’s activity by set up a Markov chain, so as to improve the sensing performed by SU. But the performance is limited because of its single threshold sensing scheme which does not consider the noise uncertainty. The performance of “Two-stage”-DE is worst among the seven kinds of algorithm since it is a sentence in Two stages, but the Two stages of the decision are dependent on energy detection and the traditional threshold calculation cannot improve the detection performance.

**Fig 6:** Performance comparison among different detection schemes.

Spectrum sensing time is one of the most important indicators of perceived performance. If the time using for spectrum sensing is too long, it is possible to improve the accuracy of detection to a certain extent. However, it can reduce users' transmission time, thereby reducing network’s throughput. Fig 7 shows the spectrum sensing time of the algorithms under different SNR when false alarm probability *P*_*f*_ = 0.1 and the samples *N =* 1000. The ADEMM needs less time compared with the other algorithms. In addition, there is a relationship between the sensing time and the SNR i.e., the sensing time decrease gradually with increase in SNR. For SNR around 20dB, the time of ADEMM needed for sensing is about 46.7ms, and for other algorithms i.e., CSBDE (*Nr* = 2), Cyclostation-DE, “Two-stage”-DE, VORDE (*Nr* = 2), ADE and ME takes about 61.2ms, 53.4ms, 61.2ms, 55.1ms, 80.8ms and 45.6ms, respectively. For false alarm probability *P*_*f*_ = 0.1, Fig 8 presents the required volume of samples to achieve the detection probability *P*_*d*_ = 0.9. It is observed that there is an inverse relationship between spectrum sensing time and SNR. As SNR decreases, the required numbers of samples increase. As compared to CSBDE, Cyclostationary-DE and “Two-stage” DE, it is observed that only few number of samples are required for AMMDE at -20dB.

**Fig 7:** The required sensing time (*P*_*f*_ = 0.1, *N* = 1000).

**Fig 8:** The required volume of samples (*P*_*f*_ = 0.1, *P*_*d*_ = 0.9).

## Discussions and conclusions

This paper introduced double-threshold energy sensing for efficient opportunity spectrum access based on Markov model and adapted the double thresholds based on the optimization function. By employing a modified Markov model, the double-threshold sensing was able to make an appropriate decision of the confused state. We analyzed the influence of noise uncertainty levels on the performance of double-threshold energy sensing. Moreover, an adaptive double-threshold method to obtain maximal objection function of probability of detection is also presented. It not only kept the sensing robustness to the noise uncertainty but also kept the sensing with a high probability of detection. The numerical simulation results showed a significant improvement in spectrum sensing efficiency as compared to the contemporary sensing schemes.

## Supporting information

S1 File Relevant data. (RAR)
